# Internet of Medical Things (IoMT) and Reflective Belief Design-Based Big Data Analytics with Convolution Neural Network-Metaheuristic Optimization Procedure (CNN-MOP)

**DOI:** 10.1155/2022/2898061

**Published:** 2022-03-18

**Authors:** A. Sampathkumar, Miretab Tesfayohani, Shishir Kumar Shandilya, S. B. Goyal, Sajjad Shaukat Jamal, Piyush Kumar Shukla, Pradeep Bedi, Meshal Albeedan

**Affiliations:** ^1^Department of Applied Cybernetics, Faculty of Science, University of Hradec Kralove, Hradec Kralove, Czech Republic; ^2^Department of Information Technology, Dambi Dollo University, Dambi Dollo, Ethiopia; ^3^School of Computing Science and Engineering, VIT Bhopal University, Bhopal, India; ^4^City University, Petaling Jaya 46100, Malaysia; ^5^Department of Mathematics, College of Science, King Khalid University, Abha, Saudi Arabia; ^6^Computer Science and Engineering Department, University Institute of Technology, Rajiv Gandhi Proudyogiki Vishwavidyalaya, (Technological University of Madhya Pradesh), Bhopal-462033, Madhya Pradesh, India; ^7^Galgotias University, Greater Noida, Uttar Pradesh, India; ^8^Department of Computer Science, Faculty of Engineering and Technology, Liverpool John Moores University (LJMU), Liverpool L3 3AF, UK

## Abstract

In recent times, the Internet of Medical Things (IoMT) is a new loomed technology, which has been deliberated as a promising technology designed for various and broadly connected networks. In an intelligent healthcare system, the framework of IoMT observes the health circumstances of the patients dynamically and responds to backings their needs, which helps detect the symptoms of critical rare body conditions based on the data collected. Metaheuristic algorithms have proven effective, robust, and efficient in deciphering real-world optimization, clustering, forecasting, classification, and other engineering problems. The emergence of extraordinary, very large-scale data being generated from various sources such as the web, sensors, and social media has led the world to the era of big data. Big data poses a new contest to metaheuristic algorithms. So, this research work presents the metaheuristic optimization algorithm for big data analysis in the IoMT using gravitational search optimization algorithm (GSOA) and reflective belief network with convolutional neural networks (DBN-CNNs). Here the data optimization has been carried out using GSOA for the collected input data. The input data were collected for the diabetes prediction with cardiac risk prediction based on the damage in blood vessels and cardiac nerves. Collected data have been classified to predict abnormal and normal diabetes range, and based on this range, the risk for a cardiac attack has been predicted using SVM. The performance analysis is made to reveal that GSOA-DBN_CNN performs well in predicting diseases. The simulation results illustrate that the GSOA-DBN_CNN model used for prediction improves accuracy, precision, recall, F1-score, and PSNR.

## 1. Introduction

In the modern world, a better healthcare system is the main challenge for the growing population of the world. The vision of the Internet of Medical Things (IoMT) is to provide a better and more pervasive health monitoring system. The IoMT is the integration of medical devices through Wi-Fi and permits device-to-device (D2D) communication. In recent days, the most challenging issue is the time needed for web services. Three-dimensional (3D) video can be downloaded at sporadic intervals by keeping in mind the latest technological trends. The collected voluminous data with less delay are obtained for accurate data measurement. It will increase the device resource allocation ability and offers quicker speed for the heterogeneous networks. The IoMT comprises various heterogeneous networks, for instance, Wi-Fi, Bluetooth, ZigBee, and other cellular platforms. The D2D communication is the central part of the IoMT platform with high efficiency and reliability. The main traits of an intelligent healthcare system are to offer less delay and high throughput and reliability, which are very important for an effective and accurate diagnosis and consultation. The critical time analysis is the key parameter to be considered for emergency healthcare applications. The highly reliable and delay-tolerant communication and transmission of data was achieved through IoT-driven wearable devices [1].

Metaheuristic optimization approaches are employed in the partitioning clustering methods with which a dataset is partitioned as groups according to the specific measure considered as a fitness function [2]. This function has a greater impact on the nature of forming these groups. When an appropriate fitness function is selected, the process of partitioning is converted as an optimization problem. Here, partitioning is performed by minimizing the distance or maximizing the similarity between the patterns, or the frequency is optimized in N-dimensional space. These techniques are generally employed in various research works as they are able to clustering large-scale datasets, like signal/image processing for segmenting images, analyzing homogeneous users to classify groups, generating precise hidden equalizers, organizing humans effectively in robotics based on their actions, matching aftershocks in seismology from background conditions, obtaining high-dimensional data report, mining web text and recognizing image patterns in computer science domain, managing portfolio in control studies, classifying diseases in medical anthropology using the medical records of patients and investigations, distributing sensor nodes in a wireless sensor network for improving lifetime, and grouping publications in library based on the contents [3].

Nowadays, big data is extensively used for analyzing the huge data for the predictors, business people, and researchers to estimate the predictions with much accuracy than the traditional analysis. Big data is structured with the five dimension maps such as velocity, value, volume, veracity, and variety. Now the researchers are working to handle scalability and the high dimension of the databases with high processing needs. Volume defines the size of the data, and velocity defines the arrival of data streams continuously from which most valuable information is gathered [4].

Moreover, in big data, the throughput, connectivity, and speed of computing have been enhanced for digital devices that improve the retrieval, progression, and fabrication of the data. Authenticity controls the information standard from different places. Variety designates the communicative path of information between different places, for example, the primary data incorporating the conventional structure. The example of data source consists of both structured traditional and relational data, along with that it also comprises of semi-structured, quasi-structured, and unstructured data such as sensor data, audio, video, text, and graph. In healthcare, big data helps in predicting epidemics, curing diseases, improving the survival rate, and avoiding unnecessary deaths. As the population in the world is increasing and the life span of individuals is long, there occur rapid changes in providing treatment, and many decisions are made based on these changes. With big data, patients take the right decision at the right time. With the data report of the patient, “proactive care” required for individuals is identified or the change required for them is analyzed so that degradation in their health can be avoided [5].

However, machine learning, as well as statistical approaches, undergoes a few necessary changes to maintain and follow some specific constraints while estimating high-dimensional data; moreover, existing issues are solved when input variables are reduced before data mining approaches are applied. Thus, there are two ways techniques are employed for dimensionality reduction in machine learning. While exploring the redundant input data or in feature selection, the essential variables are taken from the primary dataset. In the dimensionality reduction process, data are eliminated forming a new dataset with few input variables, where each column holds the combined input variables providing the same information as that of the input variables. In statistical modeling, this process is termed exploration [6]. The existing works are related to the data optimization with machine learning techniques, which does not improve the predictive accuracy with their optimization level.

The contribution of the work is as follows:

- To present the metaheuristic optimization algorithm for big data analysis in the IoMT using gravitational search optimization algorithm (GSOA) and reflective belief network with convolutional neural networks (DBN-CNNs).
- To perform data optimization using GSOA for the collected input data. The input data were collected for the diabetes prediction with cardiac risk prediction based on the damage in blood vessels and cardiac nerves.

Big data in healthcare is being used to predict epidemics, cure disease, improve quality of life, and avoid preventable deaths. With the world's population increasing and everyone living longer, the models of treatment delivery are rapidly changing, and data are driving many of the decisions behind those changes. Big data can help patients make the right decision in a timely manner. From patient data, analytics can be applied to identify individuals who need “proactive care” or need a change in their lifestyle to avoid health condition degradation. For example, patients in early stages of some diseases (e.g., heart failure often caused by some risk factors such as hypertension or diabetes) should be able to benefit from preventive care, thanks to big data.

In Section 2, the related research works are presented.  Section 3 shows the proposed model for data optimization and diabetes data classification. Evaluation criteria are discussed in Section 4. The conclusion is finally presented in Section 5.

## 2. Related Works

The healthcare system involves machine learning (ML) approaches in the fields such as diagnosing, predicting, and surveillance. It is believed by the health monitoring agents that by using ML techniques, life can be saved [7]. Using SVM, diabetic nephropathy type 2 patients can be detected [8]. Moreover, earlier detection of abnormalities can be achieved using a decision tree-based approach when integrated with genotype and clinical data of several type 2 diabetic patients. Data can be classified gender-wise using support vector machine (SVM), Naïve Bayes (NB), decision tree (DT), and random forest (RF) approaches to produce satisfactory results. In [9], ML approaches are embedded with data mining profiling for gaining knowledge from the larger collection of information. Classification approaches like SVM, NB, RF, and logistic regression (LR) are used. In [10], for cardiovascular and cerebrovascular events, an automated prediction model was developed using heart rate variability (HRV) analysis. This was suitable for patients with 55 years and more who have higher risks. 10-fold cross-validation based on HRV features with data mining approaches such as NB, DT, RF, SVM, AdaboostM1 (AB), and multilayer perceptron neural network (MLPNN) were used for prediction. Reference [11] focused on antidiabetic drug failure and developed a prediction model to maintain an exponential increase in diabetic type 2 patients. SVM was used for training large-scale medical datasets. In [12], the risk of diabetic neuropathy was examined. When diabetes has been spread in the entire body, the nervous system is affected leading to cardiac arrest. Heart rate variability (HRV) was estimated using a multiscale Allan vector and the features of ECG helped in automatic detection using ML techniques. A graph-based machine learning system (GBMLS) was introduced to diagnose diabetic neuropathy effectively. In [13], a healthy and asthma patient was comparatively examined with alternative devices to obtain the feature vector of asthma patient with the guidelines of GINA. RF, AB-RF, and MLPNN were used to develop an ML prediction model. Specificity, sensitivity, and accuracy were the parameters considered. Leave-one-out (LOO) validation methods were used to train and test the dataset to eradicate the overfitting problem. In [14], a surveillance system was introduced to effectively monitor the impacts of dengue hemorrhagic fever (DHF) and the rate of *Aedes aegypti* mosquito infection using SVM, which depends on the climate conditions and geographical area. In [15], a prediction system was designed for detecting influenza-like illness (ILI) at the earlier stages. Using NB and SVM classifiers not only produced better results but logistics regressions (LR) and sequential minimal optimization (SMO) also are suitable. In [16], an automatic coronary artery disease (CAD) diagnosis was introduced where this disease caused cardiac arrests. The diagnosis was made using tunable Q-wavelet transform (TQWT), and the heart rate signals were observed and monitored using raw ECG (electrocardiogram). With threefold cross-validation, least square support vector machine (LS-SVM) approach was used for classification. In [17], heart disease was predicted and analyzed using BagMOOV ensemble model with a multipurpose-weighted voting approach. Reference [18] studied the mood disorder which is a psychological behavior of humans and investigated a psychiatry solution using ML techniques. Three ML approaches, namely, SVM, least average shrinkage and selection operator (LASSO), and relevance vector machine (RVM) were developed using MATLAB to predict the possibilities of a suicide attempt. In [19], risks, diagnosis, and prediction of breast cancer were examined with four ML approaches, namely, SVM, DT, NB, and k-nearest neighbor (KNN). In [20], the classification of UCI's disease datasets was studied in which SVM integrated with endocrine-based particle swarm optimization (EPSO) and artificial bee bolony (ABC) was employed. In [21], it was revealed that SVM with fruit fly optimization algorithm (FOA) was used in several medical datasets, namely, Wisconsin Parkinson's dataset, breast cancer dataset, thyroid disease diagnosis, and Pima Indian diabetes dataset. In [22], a model for diabetes prediction utilizing machine learning approaches was predicted. The supervised machine learning algorithms used for the prediction model are decision tree, Naïve Bayes, artificial neural network, and logistic regression. Performance evaluation is performed in this method by employing parameters such as accuracy, recall, precision, and F1-score. In [23], the data-driven SmartWork system's AI component was described, comprising the predictive models which are personalized and decision support tools. In these subsystems, long-term predictive models and data mining techniques are implemented for providing probabilistic prediction of particular risk indicators motivated towards decision-making and T2DM intervention, among other chronic conditions.

Based on the comparison discussed, it is not enough for both optimizations to improving the accuracy. So, this research aims to propose metaheuristic algorithm for data optimization of diabetic data and the predictive analysis for cardiac attack risk prediction. Here, the IoMT module is used for data collection and uses a gravitational algorithm for data optimization, and then the data classification is done using DBN-based CNN. Finally, the predictive analysis will be done using SVM on the basis of image predictive analysis.

## 3. System Model

This section discusses the proposed metaheuristic algorithms based on data optimization for diabetes data, which leads to the predictive analysis of cardiac attack risk based on blood vessels and cardiac nerves and cardiac nerve damages. The dataset, obtained from public healthcare, contains more than 100,000 records comprising 55 attributes. Few among them are age, gender, race, number of procedures, number of medications, number of diagnoses, and readmissions.

The data have been initially collected using the IoMT module, and these data have been clustered for improving the optimization of data to be processed. Here we use metaheuristic algorithms for data optimization in which gravitational search optimization algorithm has been used. Then using these optimized data, the diabetic data have been classified for identifying the abnormal range. Here we establish a deep belief network (DBN), where the classification is carried out using CNN. By this classification, the normal range and abnormal range of diabetes have been classified. The normal diabetes range has been updated to the hospital database, and for the abnormal diabetes range, the cardiac nerve and blood vessel damages have been analyzed using SVM-based image predictive analysis. The proposed diabetic data analysis has been given in Figure 1. In the IOMT module, a dataset for diabetes is collected and the data from the dataset are clustered in the data clustering phase, and the optimization of data is done by metaheuristic data optimization by using GSOA. The optimized data are classified by the classification algorithm DBN-based CNN. From the classification results, the normal range of diabetes is sent to the hospital database, whereas an abnormal range of diabetes is sent to the analysis of predicting cardiac attack risk, which will be done by various parameters.

### 3.1. Metaheuristic-Based Gravitational Search Optimization Algorithm (GSOA)

Gravitational search optimization algorithm (GSOA) is a stochastic population-based metaheuristic approach that was developed based on Newton's laws of gravity and motion [24]. Originally, the basic GSOA model was developed to find a solution for continuous optimization problems. A set of agents/objects were introduced in the search space within dimension to determine an optimal solution where the principle of Newton's laws was followed. Here, the position of every agent describes a candidate solution *Xi*, which is a vector in the search space. An agent whose performance is higher obtains more gravitational mass as heavier objects gain more attraction radius. In the life span of GSOA, *Xi* is adjusted successively by an agent with the positions of best agents in KGSOA adapting Newton's laws. To explain in detail, a system with *s* agents is assumed, where the position of the agent is given by

(1) $$\begin{array}{c} X_{i}=\left(x_{i}^{1},\ldots ,x_{i}^{d},\ldots ,x_{i}^{n}\right);\;i=1,2,\ldots ,s, \end{array}$$

where *x*_*d*_^*i*^ represents the position of agent *i* in dimension *d* with search space dimension *n*. For every agent, the gravitational mass after estimating the current data fitness is computed as given in the following equations:

(2) $$\begin{array}{c} q_{i}\left(t\right)=\frac{{\text{fit}}_{i}\left(t\right)-\text{worst}\left(t\right)}{\text{best}\left(t\right)-\text{worst}\left(t\right)}, \end{array}$$

(3) $$\begin{array}{c} M_{i}\left(t\right)=\frac{q_{i}\left(t\right)}{\sum_{j=1}^{s}a_{j}\left(t\right)}, \end{array}$$

where *M*_*i*_(*t*) and fit_*i*_(*t*) are the gravitational mass and fitness value of *i*^th^ agent, respectively, at time *t*. The best(*t*) and worst(*t*) are given in the following equations:

(4) $$\begin{array}{c} \text{best}\left(t\right)=\min_{j\in \left(1,\ldots ,s\right)}{\text{fit}}_{j}\left(t\right), \end{array}$$

(5) $$\begin{array}{c} \text{worst}\left(t\right)={\text{max}}_{j\in \left(1,\ldots ,s\right)}{\text{f}}_{{\text{it}}_{j}}\left(t\right), \end{array}$$

Agent acceleration is estimated by adding the forces of every agent present in the set of KGSA based on the gravitational law, which is determined by using equation (6) and agent acceleration which is estimated by the motional law is expressed in equation (7):

(6) $$\begin{array}{c} F_{i}^{d}\left(t\right)=\underset{\text{jeK best,}j\neq i}{\sum }{\text{rand}}_{j}G\left(t\right)\frac{M\left(t\right)M_{i}\left(t\right)}{R_{ij}\left(t\right)+z}\left(x_{j}^{d}\left(t\right)-x_{i}^{d}\left(t\right)\right), \end{array}$$

(7) $$\begin{array}{c} a_{i}^{d}\left(t\right)=\frac{F_{i}^{d}\left(t\right)}{M_{i}\left(t\right)} \end{array}$$

where *r* and *j* are random numbers distributed evenly ranging between [0, 1],

(i) *ε*, a small value, helps to get rid of division by zero error when *R*_*ij*_(*t*) is zero.
(ii) *R*_*ij*_(*t*) represents the Euclidean distance of agents *i* and *j*, defined as kXi(*t*), Xj (*t*)k2.
(iii) *K*_best_ indicates the set of first agents in KGSOA having best fitness value and higher gravitational mass, where KGSOA is the time function which is initially assigned a *K*_initial_ value and gets decreased with time.
(iv) *G*(*t*) is the gravitational constant which initially takes *G*_initial_ value and decreases with time till *G*_end_ is reached as given in the following equation:
  (8) $$\begin{array}{c} G\left(t\right)=G\left(G_{\text{initial}},G_{\text{end}},t\right). \end{array}$$

Then, agent velocity and next position are estimated using the following equations:

(9) $$\begin{array}{c} v_{i}^{d}\left(t+1\right)={\text{rand}}_{i}*v_{i}^{d}\left(t\right)+a_{i}^{d}\left(t\right), \end{array}$$

(10) $$\begin{array}{c} x_{i}^{d}\left(t+1\right)=x_{i}^{d}\left(t\right)+v_{i}^{d}\left(t+1\right). \end{array}$$

### 3.2. Establishing DBN Architecture

Generally, when compared with a general neural network, deep neural network (DNN) is superior. In DNN, the input layer is separated from the output layer by several hidden layers. The method of training the networks differs. Particularly, in DNN, the unsupervised learning method is used for adjusting the weights in hidden layers, and the network is capable of identifying the optimal features from the input provided. Hence, DNN is flexible and enables high-order modeling of the nonlinear complex relationship between input provided to the network and output produced. The advantage of using DNN for learning the features and classifying data is proved with various pattern recognition applications like vision, speech, and natural language processing [24–26]. The outcomes observed have motivated the researchers to develop automated pattern recognition systems using DL methods. In spite of some challenges, developing a suitable training model for DNN is still a challenging one.

With the presence of several hidden layers in DNNs and numerous parameters, training has to be done with utmost care. In the process of training, the feature detection layers are randomly initialized. In DNN, a series of generative models, namely, a single visible input and a hidden layer are considered for initializing weights and are trained without taking discriminative information into account. At last, the standard back propagation approach is used to train DNN discriminatively. From the investigation, it is observed that the standard gradient-based random initialization approach used for initializing weights of the network produces very little performance in DNN containing more than two layers. As DNNs with several parameters and numerous hidden layers increase the computational complexity, training is much slower and even gets stuck with local minima providing unexpected results. Here, the parameters are initialized during unsupervised pretraining, so that the process of optimization ends with local minima of the cost function. The architecture of DBN with RBM is given Figure 2 [24].

In RBM, the energy function *E* taking parameters *v* and *h* representing a pair of visible and hidden vectors, respectively, has the general form with weight matrix *W* as in

(11) $$\begin{array}{c} E\left(v,h\right)=-a^{\tau }v-b^{\tau }h-v^{\tau }Wh, \end{array}$$

where *a* and *b* indicate the bias weights for visible and hidden units, respectively. With *v* and *h* in terms of *E*, the probability distribution *P* is given by

(12) $$\begin{array}{c} P\left(v,h\right)=\frac{1}{z}e^{-E\left(v,h\right)}. \end{array}$$

Here the normalizing constant *Z* is given by

(13) $$\begin{array}{c} Z=\underset{v^{\prime }h^{\prime \prime }}{\sum }e^{-E\left(v^{\prime }h^{\prime }\right)}\text{. } \end{array}$$

Moreover, the probability of *v* over hidden units is the sum of above given equations and is given by

(14) $$\begin{array}{c} P\left(v\right)==\frac{1}{z}\underset{h}{\sum }e^{-E\left(v,h\right)}. \end{array}$$

Log-likelihood difference of training data in terms of *W* is estimated as

(15) $$\begin{array}{c} \overset{n=N}{\underset{n=1}{\sum }}=\;\frac{\partial \text{log}P\left(v^{n}\right)}{\partial w_{ij}}\\ =v_{i}h_{j\text{data}}-v_{i}h_{j\text{model}}. \end{array}$$

where *v*_*i*_*h*_*j*data_ and *v*_*i*_*h*_*j*model_ represent the values expected for data and distribution model, respectively. For log-likelihood-based training data, network weights are computed using the learning rate *ε* as in

(16) $$\begin{array}{c} W_{ij}=\varepsilon \left(v_{i}\langle h_{j\text{data }}\rangle -\langle v_{i}h_{j\text{modea}}\rangle \right)\left(v_{i}h_{j\text{data}}\right). \end{array}$$

As neurons are not connected at either the hidden or the visible layers, it is possible to obtain unbiased samples from *v*_*i*_*h*_*j*data_. Further, the activation of hidden or visible units is conditionally independent for given *h* and *c*, respectively. For given *v*, conditional property is described in:

(17) $$\begin{array}{c} P\left(h|v\right)=\Pi_{j}\;P\left(h_{j}|v\right), \end{array}$$

where *h*_*j*_ ∈ {0,1} and the probability of *h*_*j*_=1 is given in

(18) $$\begin{array}{c} P\left(h_{j}=1|v\right)=\sigma \left(b_{j}+\underset{i}{\sum }v_{i}Wij\right). \end{array}$$

Here the logistic function *σ* is specified as in

(19) $$\begin{array}{c} \sigma \left(x\right)={\left(1+e^{-x}\right)}^{-1}. \end{array}$$

Likewise, when *v*_*i*_=1, the conditional property is estimated by

(20) $$\begin{array}{c} P\left(v_{i}=1|v\right)=\sigma \left(a_{i}+\underset{j}{\sum }W_{ij}h_{j}\;\right). \end{array}$$

Generally, with 〈*v*_*i*_, *h*_*j*_〉, the unbiased sampling is not straightforward; however, it is applicable for reconstructing the first sampling of *v* from *h* and then Gibbs sampling is used for multiple iterations. With this Gibbs sampling, every unit of the hidden and visible layers is updated in parallel. At last, with 〈*v*_*i*_, *h*_*j*_〉, the proper sampling is computed by multiplying the expected and updated values of *h* and *v*. RBM weights can be used for initializing feedforward neural networks. Among several supervised and unsupervised approaches, this work focuses on DBN as it is commonly used for classifying diabetic data.

Convolutional neural network (CNN), which is deep learning knowledge-based neural network model, is a well-described and widely used technique for classifying images. It incorporates linear convolutional layer (conv), a fully connected layer (FC), this model consists of nonlinear function with an activation function above the linear function. This nonlinear function impinges on every component of input and pooling layer and minimizes the size of the final outcomes. Multiple perceptrons are used to analyze the image inputs, and it is trained with learnable weights and bias value, which is used in several parts of images to segregate pixel values. One main advantage of using CNN is it uses a local spatial domain for the input images; in addition, it also shares a few sharable parameters and a lesser number of weights. This technique is predominately more efficient than other models due to less computation complexity and less usage of memory. The CNN architecture is shown in Figure 3 [25].

Convolutional layer: basically, the image taken as input is resized to 3 × 224 × 224, which is the standard size for the CNN model. The resized image undergoes a stack of multiple layers as convolutional layers of various receptive fields. In the convolution layer, the basic operation is a convolution where several sequential mathematical operations are performed on convoluting sliding kernel matrix over the input matrix by which feature data are extracted and then those data are mapped to the successive layers. At each co-ordinate, an element-wise matrix multiplication carries out, and the outcomes are combined to obtain a feature matrix. Convolution recurrent is a distinguishable kind of linear model that assists in various platforms such as image processing, statistics, and physics. Convolution is estimated by more than one axis. Where, two-dimensional *I* is the input image and *K* kernel filter, respectively, then the convoluted image is calculated by
  (21) $$\begin{array}{c} S\left(i,j\right)=\underset{m}{\sum }\underset{n}{\sum }I\left(m,n\right)k\left(i-m,j-n\right). \end{array}$$
Pooling layer: the pooling layer, termed also as pool, is the successive layer of the convolutional layer whose main function is to minimize the spatial domain representation thereby reducing the network computations performed. Generally, in CNN, the pooling kernel is 2 × 2 in size with a stride of 2.
Fully connected layer: this FC layer is replicated in CNN due to convolution. *n*1 × *n*2 is its usual size, where *n*1 and *n*2 are the size of the input tensor (7 × 7 × 512) and output tensor, respectively, which is normally an integer.
Dropout: this layer is abbreviated as “Drop.” Usually, it is employed for eliminating the input overfits; the basic role is to improve the conjecture of deep learning methods. Normally, it assigns the weights to the connected network nodes.
Softmax: normally represented as “*σ*,” is a deep learning model followed by many layers and the convolutional layer is followed by a ReLU layer which determines the nonlinearity of CNN and improves it.

The convolution layers present within both the pooling layers possess the equal channel number, kernel size, and stride. Actually, collecting two 3 × 3 convolution layers and three 3 × 3 convolution kernels is equal to a single 5 × 5 and 7 × 7 convolution layers, respectively. Stacking 2 or 3 small convolution kernels works much quicker than a single huge convolution kernel. Moreover, parameter numbers have been minimized. ReLU layers, which are inserted among undersized convolution layers, are really useful.

The input data and their corresponding map images are *S* = (S ^(1)^ … S ^(*N*)^) and *M* = (M ^(1)^ … *M*^(*N*)^), respectively. The major objective is to design a model which maps *S* to *M* with the help of some training data. This is modeled as a probabilistic approach by learning the model of distribution over labels which is represented by

(22) $$\begin{array}{c} P\left(n\left(M,i,w_{m}\right)|n\left(S,i,w_{s}\right)\right), \end{array}$$

where *n* (*I*, *i*, *w*) is a patch with *w* ∗ *w* size for image *I,* focused on pixel *i*. Here, *W*_*S*_*W*_*S*_ is preferred to be higher so that more contextual information can be extracted. Its functional form *f* is given by

(23) $$\begin{array}{c} f_{t}\left(s\right)=\sigma \left(a_{1}\left(s\right)\right)\\ =P\left(m_{1}=\frac{1}{s_{1}}\right), \end{array}$$

where *a*_*i*_ and *f*_*i*_ represent the sum of input for the *i*^th^ output and significance of *i*^th^ output component, respectively. (*x*), a logistic utility, is expressed by

(24) $$\begin{array}{c} \left(x\right)=\frac{1}{1+\text{exp}\left(-x\right)}. \end{array}$$

CNN alongside softmax output unit is used for multiclass marking. The softmax output is a vector of size *L*, which demonstrates the conveyance more than potential marks for pixel *i*. Along these lines for multiclass marking, if the path from pixel *i* to output unit *l* is thought of, the recomposed condition is given in

(25) $$\begin{array}{c} f_{il}\left(s\right)=\frac{\text{exp}\left(a_{il}\left(S\right)\right)}{z}\\ =P\left(m_{i}=l|s\right), \end{array}$$

where *f*_*il*_(*s*) is the prediction probability, where pixel *I* is mapped to label *j*. The advantages of the proposed method are summarized as follows:

- First, CNN possibly handles a huge amount of labelled data from various domains.
- Second, it is faster when paralleled with graphics processing unit (GPU). Hence this is also extended for a greater number of pixels. The kernel size has been minimized to simulate the training data, and the kernel size minimization is performed by the computational learning process of the proposed method.
- Every patch in training data has been given by initiative sigma. Due to a large number of training patches, optimization becomes complicated. This can be done using a binary classifier that uses minimum patches. Few of the hyper parameters have been altered to some extent. The analysis over sensitivity has been defined by hyper parameters for them to be tuned with higher accuracy.

The output from the softmax layer will be classified to be normal and abnormal ranges of diabetes, and the abnormal range of diabetes will be carried out for the predictive analysis of cardiac attack based on the cardiac nerve and blood vessel damage. This has been analyzed by using SVM-based image predictive analysis.

### 3.3. SVM-Based Image Predictive Analysis

SVM method is employed in classification and regression. With methods based on SVM, data points with identical properties are grouped together depicting the space. With linear SVM, for the data provided, p-dimensional vector is contemplated and divided by utmost p-1 planes called hyperplanes, which are employed to divide the space for classification and regression. The mathematical form of SVM is given. The line equation is outlined by

(26) $$\begin{array}{c} a_{1}=a_{2}x+b. \end{array}$$

In (26), “*x*” stands for the line's slope and “*b*” stands for intersect as given in

(27) $$\begin{array}{c} a_{1}-a_{2}x+b=0. \end{array}$$

Let *a*′=(*a*_1_, *a*_2_)^*T*^ and *z*′=(*x*, −1). Thus,

(28) $$\begin{array}{c} z^{\prime }.a^{\prime }+=0. \end{array}$$

The above equation obtained from two-dimensional vectors is known as the hyper lane equation. *a*′=(*a*_1_, *a*_2_)^*T*^ is mentioned as *z*′ as given in

(29) $$\begin{array}{c} z^{\prime }=\frac{a_{1}}{\left\|a\right\|}+\frac{a_{2}}{\left\|a\right\|}. \end{array}$$

Here,

(30) $$\begin{array}{c} \left\|a\right\|=\sqrt{a_{1}^{2}+a_{2}^{2}+a_{3}^{2}+\cdots \cdot a_{n}^{2}}. \end{array}$$

It is known that

(31) $$\begin{array}{c} \text{cos}\left({\text{g}}_{1}\right)=\frac{a_{1}}{\left\|a\right\|},\\ \text{coscos}\left({\text{g}}_{2}\right)=\frac{a_{2}}{\left\|a\right\|}. \end{array}$$

Moreover, this can be expressed as equations (32)–(35):

(32) $$\begin{array}{c} z^{\prime }=\left(\cos\cos\left(I_{1}\right),\;\cos\cos\left(U_{2}\right)\right), \end{array}$$

(33) $$\begin{array}{c} z^{\prime }\cdot a=\left\|z\right\|\left\|a\right\|\text{cos}\left(\theta \right), \end{array}$$

(34) $$\begin{array}{c} \theta =\theta_{1}-\theta_{2}, \end{array}$$

(35) $$\begin{array}{c} z^{\prime }\cdot a^{\prime }=\overset{n}{\underset{i=1}{\sum }}z_{i}^{\prime }a_{i}. \end{array}$$

For *n*-dimensional vectors, dot product is computed as follows: consider *f* = *y*(*z*…*a* + *b*) when sign (*f*) > 0, then it is a correct categorization, and for sign (*f*) < 0, it is incorrect. If dataset *D* is provided, then on a training dataset, *f* is calculated by

(36) $$\begin{array}{c} f_{i}=y_{i}\left(z^{\prime }\cdot a+b\right). \end{array}$$

Functional margin (*F*) on the dataset is estimated as given in

(37) $$\begin{array}{c} F={\text{min}}_{i=1\ldots m}f_{i}. \end{array}$$

Through the contrast between the hyperplanes, hyperplane having greatest *F* is chosen. For selecting optimal hyperplane, optimal *z* and *b* values have to be found. Lagrangian function *L* is given by the following equations:

(38) $$\begin{array}{c} L\left(z^{\prime },b,\alpha \right)=\frac{1}{2}z^{\prime }\cdot z^{\prime }-\overset{m}{\underset{i=1}{\sum }}\alpha_{i}\left[y:\left(z^{\prime }\cdot a+b\right)-1\right]\text{,} \end{array}$$

(39) $$\begin{array}{c} {}_{b}L\left(z^{\prime },b,\alpha \right)=-\overset{m}{\underset{i=1}{\sum }}\alpha_{i}y_{i}=0. \end{array}$$

Thus *z*′ is calculated as follows:

(40) $$\begin{array}{c} z^{\prime }=\overset{m}{\underset{i=1}{\sum }}\alpha_{i}y_{i}a_{i},\\ \overset{m}{\underset{i=1}{\sum }}\alpha_{i}y_{i}=0.\; \end{array}$$

In the following equation, replacing *L*,

(41) $$\begin{array}{c} z^{\prime }\left(\alpha ,b\right)=\overset{m}{\underset{i=1}{\sum }}\alpha_{i}-\frac{1}{2}\overset{m}{\underset{i=1}{\sum }}\overset{m}{\underset{i=1}{\sum }}\alpha_{i}\alpha_{j}y_{i}y_{j}a_{i}a_{j}. \end{array}$$

Thus, the following equation is obtained:

(42) $$\begin{array}{c} {\text{max}}_{\alpha }=\overset{m}{\underset{i=1}{\sum }}\alpha_{i}-\frac{1}{2}\overset{m}{\underset{i=1}{\sum }}\overset{m}{\underset{i=1}{\sum }}\alpha_{i}\alpha_{j}y_{i}y_{j}a_{i}a_{j}. \end{array}$$

When a point lies over the hyperplane, it is categorized as +1 class describing those cardiac risks are identified while under the hyperplane, it is −1 class describing that no cardiac risks are identified.

## 4. Performance Analysis

For the performance evaluation of the proposed method, MATLAB software is used for implementation. The efficiency of the proposed method is evaluated with a few parametric measures like accuracy, precision, recall, and F1-score. By using the U-matrix error rate of topographical error, then quantization error has been estimated. The dataset chosen for estimation is the diabetic dataset. To test the performance of the model, data are randomly selected from the dataset.

### 4.1. Quantization Error

During training, the required amount of computation level is reduced. Moreover, it estimates the performance level by applying stochastic quantization evaluating the value of the gradients. It regulates the standard distance between every input vector of the node and its winner.

(43) $$\begin{array}{c} Q_{e}=\frac{1}{N}\overset{N}{\underset{j=1}{\sum }}\left|\left|x_{j}-w_{j}\right|\right|. \end{array}$$

In the above equation, *w*_*j*_ indicates the weight vector of winner for input *x*_*j*_. Thus, the expected *Q*_*e*_ has to be small.

### 4.2. Neuron Utilization *N*_*U*_

This specifies the ratio of the winner neurons of a single input or more inputs in vector map.

(44) $$\begin{array}{c} N_{U}=\frac{1}{nm}\overset{mm}{\underset{i=1}{\sum }}u_{i}. \end{array}$$

Here by (45), if neuron *i* is the winner, then *u*_*i*_=1 or *u*_*i*_=0. Therefore, *N*_*U*_ closer to 1.0 is more expected. The error calculation is shown in Figures 4(a) and 4(b)

### 4.3. U-Matrix

The U-matrix represents the cluster structure of the map illustrating the distances of the adjacent neurons. Output classes of the winning neurons of the U-matrix and winning neurons with class names are shown in Figures 5(a) and 5(b)

### 4.4. Accuracy

This gives the ratio of the instances classified correctly which is estimated by

(45) $$\begin{array}{c} \text{accuracy rate}=\frac{\text{true positive}+\text{true negative}}{\text{total instances}}*100. \end{array}$$

### 4.5. Precision

This is the measure which reveals the ratio of data transmitted in the network with intrusion. This parameter estimates the correctness and quality of classification which is determined by

(46) $$\begin{array}{c} \text{precision}=\frac{\text{true positive}}{\text{true positive}+\text{false positive}}. \end{array}$$

### 4.6. Recall

This metric presents the proportion of real positives that are correctly predicted positives given by

(47) $$\begin{array}{c} \text{recall}=\frac{\text{true positive}}{\text{true positive}+\text{false positive}}. \end{array}$$

### 4.7. F1-Score

This is generally the mean value of precision and recall. Moreover, statistical measure is used in F1-score to calculate the performance rate of individual classifier of FN and FP as given in (49). Precision judges the accuracy, while recall detects sample instances with respect to faulty or nonfaulty attributes.

(48) $$\begin{array}{c} F1\text{ score}=\frac{2X\text{precision}\times \text{recall}}{\text{precision}+\text{recall}}. \end{array}$$

Table 1 shows some of the observations from the instances of diabetic datasets, which are then classified. The performance measures of various techniques of KNN, NN, and ANN are considered for estimating the efficiency of the proposed GSOA-DBN_CNN technique. Table 1 presents the comparative analysis of accuracy, precision, recall, and F1-score, which are represented in percentage.

Figure 6 graphically represents the comparison for various methods in terms of accuracy. It is observed that the proposed GSOA-DBN_CNN technique produced more accuracy than the existing techniques. Accuracy has been improved for proposed technique as 98%.

Figure 7 graphically represents the comparison for various methods in terms of precision. It is proved that the proposed GSOA-DBN_CNN technique produced higher precision than the existing techniques. By comparing precision analysis with existing technique, the proposed technique has been improved as 96%.

Figure 8 graphically represents the comparison for various methods in terms of recall. It is noticed that the proposed GSOA-DBN_CNN technique produced maximum recall than the existing techniques. Recall has been improved as 94% for proposed technique when compared with existing technique.

Figure 9 graphically represents the comparison for various methods in terms of F1-score. It is discovered that the proposed GSOA-DBN_CNN technique achieves improved F1-score as 92% than the existing techniques.

PSNR graph comparison for proposed GSOA and existing ACO, WOA, GA, and HA is shown in Figure 10.

Figure 10 graphically represents the comparison for various methods in terms of PSNR comparison for data optimization. It is inferred that the proposed GSOA-DBN_CNN technique achieves improved 0.2 PSNR than the existing techniques.

The comparative results are described in the Table 2, and the overall analyses show that the proposed GSOA-DBN_CNN achieved accuracy higher than 2% of ANN, 3% of NN, and 4% of KNN. The precision achieved is more than 2% of ANN, 3% of NN, and 6% of KNN. Recall obtained is higher than 2% of ANN, 3% of NN, and 4% of KNN, similarly the F1-score achieved is 2% of ANN, 3% of NN, and 3% of KNN. The proposed GSOA-DBN_CNN technique achieves improved 0.2 PSNR than the existing AWO, WOA, and GA techniques which is shown in Figure 11.

From the experimental results, it is observed that the proposed GSOA-DBN_CNN technique achieves accuracy of 98%, 96% of precision, recall of 94%, and PSNR of 0.2 higher than the existing ACO, WOA, and GA techniques. Although the proposed GSOA-DBN_CNN model achieves better results, it lacks efficiency in some areas, which is to be improved.

## 5. Conclusion

The efficiency of the metaheuristic optimization algorithms is proved by solving several issues related to text clustering. But, the trapping of local optima is possible as the focus is on global search rather than on local search, that is exploration instead of exploitation. In this study, a metaheuristic algorithm based on data optimization is proposed for diabetes data, which leads to the predictive analysis of cardiac attack risk based on blood vessels and cardiac nerves and cardiac nerve damages. For data optimization, GSOA is used since those metaheuristic optimization algorithms are robustly feasible. Then, a deep belief architecture (DBA) is established, where the classification is carried out using CNN. By this classification, the normal range and abnormal range of diabetes have been classified. The normal diabetes range has been updated to the hospital database, and for the abnormal diabetes range, the cardiac nerve and blood vessel damages have been analyzed using SVM-based image predictive analysis. Further, the method has also been compared with ACO, WOA, GA, and HA. The results reveal that the proposed GSOA-DBN_CNN technique is better in terms of every parameter considered for comparison against the existing techniques. The accuracy achieved by the proposed technique is 98%, precision attained is 96%, the recall has been improved up to 94%, and F1-score obtained by 92% when compared with existing KNN, ANN, and NN. The comparative results are described as follows: the proposed GSOA-DBN_CNN achieved accuracy higher than 2% of ANN, 3% of NN, and 4% of KNN. The precision achieved is more than 2% of ANN, 3% of NN, and 6% of KNN. Recall obtained is higher than 2% of ANN, 3% of NN, and 4% of KNN, similarly, the F1-score achieved is 2% of ANN, 3% of NN, and 3% of KNN. The proposed GSOA-DBN_CNN technique achieves an improved 0.2 PSNR than the existing AWO, WOA, and GA techniques. The data optimization has been improved when compared with existing optimization techniques in terms of PSNR. In the future, hybrid deep learning methods can be utilized to further improve the efficiency of the model.

## Figures and Tables

**Figure 1:** Proposed design for metaheuristic algorithms for data optimization with the IoMT.

**Figure 2:** Architecture of the DBN with RBM.

**Figure 3:** Architecture of the convolutional neural network.

**Figure 4:** (a) Quantization error calculation and (b) topographic error calculation.

**Figure 5:** (a) Output classes of the winning neurons of the U-matrix and (b) winning neurons with class names.

**Figure 6:** Comparison of accuracy.

**Figure 7:** Comparison of precision.

**Figure 8:** Comparison of recall.

**Figure 9:** Comparison of F1-score.

**Figure 10:** PSNR comparison for data optimization.

**Figure 11:** Overall comparison.

**Table 1:** Comparison of performance.

Parameters	KNN	NN	ANN	GSOA-DBN_CNN
Accuracy	94	96	97	98
Precision	89	92	94	96
Recall	87	88	91	94
F1-score	82	86	88	92

**Table 2:** Overall result comparison.

Algorithm	Accuracy (%)	Precision (%)	Recall (%)	F1-score (%)
KNN	94	92	90	88
NN	95	95	91	88
ANN	96	96	92	90
GSOA-DBN_CNN	98	98	94	92

## Data Availability

The data used to support the findings of this study are included within the article.
